The article "Curcumin Alleviates D-Galactose-Induced Cardiomyocyte Senescence by Promoting Autophagy via the SIRT1/AMPK/mTOR Pathway" was published in 2022. Journal: Evid Based Complement Alternat Med.

# Curcumin Alleviates D-Galactose-Induced Cardiomyocyte Senescence by Promoting Autophagy via the SIRT1/AMPK/mTOR Pathway

**DOI:** 10.1155/2022/2990843

**Published:** 2022-07-16

**Authors:** Lei Yang, Jun Shi, Xiaowan Wang, Rong Zhang

**Affiliations:** ^1^Department of Geriatrics, Xinhua Hospital Affiliated to Shanghai Jiaotong University School of Medicine, Shanghai 200092, China; ^2^Department of Emergency, Shanghai General Hospital, Shanghai Jiao Tong University School of Medicine, Shanghai 200080, China; ^3^Department of Cardiology, Shi Dong Hospital Affiliated to University of Shanghai for Science and Technology, 999 Shiguang Road, Shanghai 200438, China; ^4^Department of Emergency, Xinhua Hospital Affiliated to Shanghai Jiaotong University School of Medicine, Shanghai 200092, China; ^5^Department of Nephrology, Shanghai General Hospital, Shanghai Jiao Tong University School of Medicine, 100 Haining Road, Shanghai 200080, China

## Abstract

Oxidative stress and impaired autophagy are the hallmarks of cardiac aging. However, there are no specific drugs available to prevent cardiac aging. Curcumin is a natural polyphenolic drug with antioxidant, antiaging, and autophagy-promoting effects. Here, we describe the preventive role of Curcumin in cardiac aging through the induction of autophagy and the restoration of autophagy via the SIRT1/AMPK/mTOR pathway. The number of cells positive for senescence-associated *β*-galactosidase, P53, P16, and intracellular ROS increased significantly in senescent cardiomyocytes, stimulated using D-galactose. Curcumin reversed this effect in a dose-dependent manner. Curcumin-induced autophagy increased the expression of SIRT1and phosphorylated AMPK and decreased phosphorylated mTOR in a dose-dependent manner. SIRT1-siRNA-mediated knockdown inhibited the antioxidation, antiaging, the promotion of autophagy, and the SIRT1/AMPK/mTOR pathway activation effect of curcumin. Therefore, curcumin could be an effective anticardiac aging drug.

## 1. Introduction

Aging is a prominent independent risk factor for the cardiovascular disease (CVD) [1], which is the most prevalent disease with the highest morbidity and mortality worldwide [2]. Global aging trends necessitate the development of new interventions focused on the treatment and prevention of heart diseases. Understanding the underlying cellular and molecular pathogenesis of cardiac aging is critical for developing interventions for CVDs in the elderly [3]. Increased oxidative stress, misfolded and denatured proteins, mitochondrial dysfunction, and impaired autophagy are the primary molecular and cellular changes during cardiac aging [4].

A hallmark of cardiac aging is mitochondrial dysfunction, which subsequently leads to excessive reactive oxygen species (ROS) and oxidative stress [5]. Excessive oxidative stress induces subcellular organelle damage, especially in the mitochondria, and causes protein aggregation [6]. Additionally, oxidative stress alters cascades in the signaling pathways involved in aging and autophagy. Therefore, oxidative stress contributes to cardiac aging [7]. Cardiomyocytes cannot replicate, however, they are metabolically active. Therefore, the intracellular renewal mechanisms, especially autophagy, is essential for maintaining the homeostasis in cardiomyocytes [8].

Autophagy is a fundamental cellular process through which molecules and subcellular components are degraded via the lysosomal pathway. The products are recycled [9]. Autophagy is critical for the maintenance of cellular homeostasis [10]. Autophagy is inhibited in the aging heart. It involves various molecular pathways, such as mTORC1, AMPK, Sirtuins, FoxO, TFEB, and ROS [11]. There is also an interaction between ROS and autophagy. The mitochondria, endoplasmic reticulum, peroxisomes, and proteins damaged by oxidative stress are degraded and recycled through autophagy to slow cell death. A moderate amount of ROS can induce autophagy, however, excessive ROS inhibits autophagy and aggravates protein aggregation and mitochondrial function damage, contributing to the increased generation of ROS, forming a vicious circle. Interventions that modulate autophagy and oxidative stress could reverse cardiac aging. However, they are difficult to characterize.

The polyphenolic compound curcumin is derived from turmeric and possesses therapeutic and biological properties against many human health issues [12]. Experiments *in vitro* and *in vivo* suggest that curcumin could prevent cardiovascular diseases, alleviate cardiovascular aging, and induce autophagy via various signaling pathways, including SIRT, AMPK, and mTOR [13]. Curcumin has antioxidant, autophagy-promoting, and antiaging properties. Therefore, we hypothesized that curcumin could be a potential anticardiac aging agent. However, further investigation into the intrinsic mechanism of the pharmacological action of curcumin is needed.

Curcumin activates AMPK and suppresses mTOR signaling pathways in an ischemia-induced cardiomyocyte injury model [14]. mTOR and the regulatory-associated protein of mTOR (Raptor), which negatively regulate autophagy by phosphorylating ULK1, form mTOR complex 1 (mTORC1), which is an essential kinase for the initiation of autophagy. The AMPK pathway controls autophagy by directly activating ULK1 or inhibiting mTORC1 [15].

Sirtuins (SIRT) are NAD^+^-dependent deacetylases that are highly conserved between yeast and humans. SIRT1 is the most broadly investigated member of this family [16]. SIRT1 plays a positive role in autophagy and longevity and can activate AMPK/mTOR signaling in different pathologies [17]. SIRT1 can be induced by curcumin. Therefore, we hypothesized that curcumin ameliorates D-galactose-induced cardiomyocyte senescence by promoting autophagy, subsequently reducing the oxidative stress in cardiomyocytes. To test this hypothesis, we treated cardiomyocytes with D-galactose (10 g/l, 48 h) to develop a senescent cell model induced by oxidative stress. The cells were treated with different concentrations of curcumin. Senescence-associated *β*-galactosidase (SA-*β*-gal) staining, DCFH-DA staining, mRFP-GFP-LC3 staining, and western blotting were used to assess the effects of Curcumin in terms of autophagy, oxidative stress, and senescence. siRNA-mediated SIRT1 knockdown was used to identify the possible signaling pathways affected by curcumin.

## 2. Materials and Methods

### 2.1. Cell Culture and Treatment

Primary neonatal rat cardiomyocytes were obtained from Sprague-Dawley (SD) rats aged 1–2 days (Jihui Animal Experiment Company, Shanghai, China). Animal research was approved by the Animal Care Committee of the Animal Experimental Center, Xinhua Hospital, Shanghai Jiao Tong University School of Medicine (Shanghai, China). The hearts were cut into pieces and digested with 0.08 trypsin (Gibco, USA) for 16–20 h at 4°C. Following the termination of the digestion, we added 0.06% collagenase II (Worthington, USA) and incubated the cells at 37°C (3–4 times for 10 min each). After all the tissue blocks were completely digested, we collected cells by centrifugation at 4°C for 10 min at 1000 rpm. The cells were incubated at 37°C at 5% CO_2_ for 2 h. The fibroblasts were attached to the dishes. The unattached cardiomyocytes were recultured in a new medium containing 10% calf serum, 1% penicillin and streptomycin, and DMEM (Gibco, USA). In addition, 5-bromo-2-deoxyuridine (0.1 mmol/l; Sigma) was added to exclude cardiac fibroblasts. After 72 h, most cells adhered to the surface of the culture dishes. The cells were treated with D-galactose (10 g/l) (Sigma, USA) for 48 h to establish the cardiomyocyte aging model [18]. The cells were then treated with curcumin at 1 *μ*M, 5 *μ*M, or 10 *μ*M in the medium containing D-galactose (10 g/L).

### 2.2. Senescence-Associated *β*-Galactosidase Assay

Senescent cardiomyocytes were assessed using a senescence-associated *β*-galactosidase (SA-*β*-gal) staining kit (Cell Signaling Technology, USA). The cells were washed with phosphate-buffered saline three times. They were fixed for 15 min in a fixative solution at room temperature and then incubated overnight with a staining solution mix at 37°C. Senescent cells (SA-*β*-gal-positive) were identified under a microscope as blue-stained cells.

### 2.3. Western Blotting

The cardiomyocytes were lysed using a buffer (RIPA with phosphatase inhibitor, Beyotime Biotechnology, China). An Enhanced BCA Protein Assay Kit (Beyotime Biotechnology, China) was used to quantify protein concentrations. The samples were diluted to standardize the protein concentration. The proteins were separated using sodium dodecyl sulfate-polyacrylamide gel electrophoresis (SDS-PAGE) and then transferred to polyvinylidene difluoride (PVDF) membranes. The membranes were cut according to the molecular weight of the proteins, and they were blocked with blocking buffer (5% non-fat dry milk in PBST) for 1 h, following which, the membranes were incubated with specific antibodies overnight at 4°C. The membranes were washed three times with TBST and incubated with a secondary antibody labeled with horseradish peroxidase (1 : 5000; Abclonal, China) at room temperature for 1 h. The primary rabbit antibodies included mTOR (1 : 1000; Cell Signaling Technology, USA), phospho-mTOR (1 : 1000; Cell Signaling Technology, USA), AMPK (1 : 1000; Cell Signaling Technology, USA), phospho-AMPK (1 : 1000; Cell Signaling Technology, USA), SIRT1 (1 : 1000; Cell Signaling Technology, USA), P53 (1 : 500; Abclonal, China, A19585), P16 (1 : 2000; Abcam, USA), LC3I/II (1 : 2000; Abcam, USA), P62 (1 : 1000; Cell Signaling Technology, USA), and GAPDH (1 : 1000; Cell Signaling Technology, USA). The immunoreactive proteins were observed using the enhanced chemiluminescence method (ECL) with Millipore's electroluminescent solution (USA) and analyzed using ImageJ (USA).

### 2.4. Detection of Reactive Oxygen Species (ROS)

To detect intracellular ROS, we used a reactive oxygen species assay kit (Beyotime Biotechnology, China). DCFH-DA is nonfluorescent, however, intracellular esterases hydrolyze it to generate DCFH after it enters the cell. Reactive oxygen species in the cell oxidizes the nonfluorescent DCFH to produce fluorescent DCF. The DCF fluorescence can be used to determine the level of intracellular reactive oxygen species. The cells were incubated with 10 *μ*mol/L DCFH-DA for 30 min at 37°C, washed thrice with DMEM, and observed immediately under a fluorescence microscope and analyzed using ImageJ.

### 2.5. mRFP-GFP-LC3 Staining

To analyze autophagy flux, we treated cardiomyocytes with fluorescent-tagged RFP-GFP-LC3 adenovirus (Shanghai hanheng Biotechnology, China) for 24 h. The cardiomyocytes were then treated with D-gal and curcumin for 48 h for subsequent assays. The cells were observed under a fluorescence microscope and analyzed using ImageJ software.

### 2.6. siRNA-Mediated SIRT1 Knockdown

Short interfering RNA (siRNA) was used to knockdown rat SIRT1. The siSIRT1 and control siRNA were purchased from Shanghai Hanheng Biotechnology (Shanghai, China). Cardiomyocytes were seeded into six-well plates and cultured until they reached 70–80% confluence. They were transfected with siSIRT1 and control siRNA using HiPerFect (Qiagen, USA) and cultured for 24 h. The cells were then treated with D-gal and curcumin for 48 h for subsequent assays.

### 2.7. Statistical Analysis

Statistical analyses were conducted using GraphPad Prism 9.0 program. The results are expressed as mean ± standard deviation (SD). We analyzed the data using one-way ANOVA. Significance was set at *P* < 0.05.

## 3. Results and Discussion

### 3.1. Curcumin-Inhibited Senescence and Oxidative Stress in D-Galactose-Induced Senescent Cardiomyocytes

To explore whether curcumin has protective effects against aging and oxidative stress in cardiomyocytes, we induced senescence in primary rat cardiomyocytes by treating them with D-galactose (10 g/l) for 48 h. D-galactose is commonly used to establish an aging model through the induction of oxidative stress. We evaluated two age-related parameters: senescence-associated-*β*-galactosidase (SA-*β*-gal) activity and the expression of P53 and P16 proteins. There was a remarkable increase in SA-*β*-gal stain-positive cells among the cardiomyocytes treated with D-galactose without curcumin. However, curcumin treatment reversed these effects in a dose-dependent manner (Figures 1(a) and 1(b)). A marked increase in the expression of p53/p16 was observed in D-galactose-induced senescent cardiomyocytes. It was suppressed by curcumin in a dose-dependent manner (Figures 1(c), 1(d), and 1(e)). Therefore, curcumin alleviated senescence in D-galactose-induced senescent cardiomyocytes.

To determine whether curcumin could attenuate oxidative stress in senescent cardiomyocytes, we assessed the level of intracellular ROS in cardiomyocytes using DCFH-DA. Consistent with the results of the two age-related parameters, DCFH-DA-positive cells were notably higher in senescent cardiomyocytes, and it gradually reduced under curcumin treatment in a dose-dependent manner (Figures 1(f) and 1(g)). Therefore, curcumin attenuated oxidative stress in senescent cardiomyocytes.

### 3.2. Curcumin Promoted Autophagy in D-Galactose-Induced Senescent Cardiomyocytes

Western blot analysis was used to assess the levels of proteins associated with autophagy to determine whether curcumin improves cardiac aging by promoting autophagy. The levels of the unique markers, LC3 II/I and p62, were assessed. The LC3 II/I ratio decreased notably following the D-galactose treatment. It increased with curcumin treatment in a dose-dependent manner (Figures 2(a)–2(c)). In contrast, p62 protein levels significantly increased in the D-galactose treatment. Curcumin reversed this trend in a dose-dependent manner. Cardiomyocytes were infected with a GFP-mRFP-LC3 fluorescent protein-expressing adenovirus to determine the role of curcumin in an autophagic flux. RFP is insensitive to acid, while GFP is sensitive to acid. Therefore, when an acidic autolysosome is formed, GFP green fluorescence is quenched. Therefore, we observed the transition from autophagosomes to autolysosomes under a fluorescence microscope. The D-galactose treatment attenuated both red fluorescent protein (RFP) and green fluorescent protein (GFP) signals. Yellow spots indicating a merge of green and red fluorescence, representing autophagosomes, were observed. Therefore, D-galactose treatment inhibited the formation of autolysosomes and autophagosomes. However, curcumin treatment facilitated the formation of autolysosomes and autophagosomes (Figures 2(d) and 2(e)). Therefore, curcumin promoted autophagy in senescent cardiomyocytes.

### 3.3. Curcumin-Enhanced SIRT1/AMPK/mTOR in D-Galactose-Induced Senescent Cardiomyocytes

To determine whether SIRT1/AMPK/mTOR is a potential pathway influenced by curcumin, we measured the total and phosphorylated levels of AMPK, mTOR, and SIRT1. The levels of SIRT1 and phosphorylated AMPK were notably decreased by D-galactose treatment but were reversed by curcumin treatment in a dose-dependent manner (Figures 3(a), 3(c), and 3(d)). The phosphorylation of mTOR increased significantly by the induction of cardiomyocytes with D-galactose and was suppressed following the addition of curcumin in a dose-dependent manner. Therefore, curcumin might induce autophagy through the SIRT1/AMPK/mTOR signaling pathway.

### 3.4. siSIRT1 Blocked the Anti-Aging Effects and Antioxidant Effect of Curcumin in D-Galactose-Induced Senescent Cardiomyocytes

Curcumin improves myocardial senescence and reduces intracellular ROS by inducing the SIRT1/AMPK/mTOR pathway. Therefore, we suppressed SIRT1 gene expression by siRNA-mediated knockdown. The knockdown of SIRT1 blocked the antiaging effects of curcumin in D-galactose-induced senescence (Figures 4(a), 4(b), 4(c), 4(d), and 4(e)), compared to that in the group transfected with control siRNA. The group transfected with siSIRT1 had a higher number of senescence-*β*-galactosidase-positive cells. p53 and p16 protein levels were considerably higher in the SIRT1 knockdown groups. SIRT1 gene knockdown blocks curcumin's antioxidant effect in D-galactose-induced senescence (Figures 4(f) and 4(g)). DCFH-DA positive cells were notably higher in the SIRT1 gene knockdown groups. In summary, knockdown with siSIRT1 blocked the antiaging and antioxidant effects of curcumin in D-galactose-induced cardiomyocyte senescence. Therefore, curcumin promoted autophagy by enhancing the SIRT1/AMPK/mTOR pathway in D-galactose-induced senescent cardiomyocytes.

### 3.5. siSIRT1 Inhibited the Facilitation of Autophagy by Curcumin in D-Galactose-Induced Senescent Cardiomyocytes

To determine whether curcumin promotes autophagy through the SIRT1/AMPK/mTOR pathway, we used siSIRT1 to block the expression of SIRT1. Compared to the NC group, the LC3 II/I ratio decreased in both SIRT1 knockdown groups. However, the p62 expression increased (Figures 5(a), 5(b), and 5(c)). The red fluorescent protein (RFP) signal weakened in the siSIRT1-treated groups. However, yellow spots were observed, revealing the restrained formation of autolysosomes and autophagosomes. Therefore, siSIRT1 inhibited the autophagy-promoting effect of curcumin in senescent cardiomyocytes induced by D-galactose.

### 3.6. siSIRT1 Inhibited the Promotion of the SIRT1-AMPK/mTOR Pathway by Curcumin

We evaluated the effect of siSIRT1 on the expression levels of SIRT1, total and phosphorylated AMPK, and mTOR. The expression of SIRT1((Figures 6(a) and 6(b)), and the levels of phosphorylated AMPK ((Figures 6(a) and 6(c)) were decreased in the SIRT1 knockdown groups relative to that in the control siRNA treated groups. However, the levels of the phosphorylated mTOR protein ((Figures 6(a) and 6(d)) increased. Therefore, siSIRT1 treatment inhibited the effect of curcumin on the SIRT1/AMPK/mTOR pathway.

## 4. Discussion

Curcumin promoted autophagy by positively regulating the SIRT1/AMPK/mTOR pathway to alleviate intracellular oxidative stress and subsequently delay aging. It could be attributed to the following reasons: excessive oxidative stress induced by D-galactose attenuates the SIRT1/AMPK/mTOR pathway, inhibits autophagy, and promotes cellular senescence. Curcumin application enhanced the SIRT1/AMPK/mTOR pathway, markedly augmented autophagy, reduced oxidative stress, and attenuated cellular senescence. The autophagy-promoting, intracellular ROS-lowering, and AMPK/mTOR pathway-promoting effects were inhibited after the knockdown of SIRT1 using siRNA.

Oxidative stress, an imbalance between oxidative and antioxidative systems, is a hallmark of cardiac aging [19]. Excessive ROS causes oxidative damage, including DNA mutations, protein oxidation, and damage to ion channels and organelles, disrupting the homeostasis of the internal environment and contributing to cardiac aging [20].

Impaired autophagy is another hallmark of cardiac aging. In mice, Atg5-deficiency causes cardiomyopathy associated with progressive aging [21]. ATG5 expression prolongs the lifespan of mice through autophagy [22]. The disruption of Beclin1-Bcl2, an inhibitor of membrane nucleation, promotes autophagy, slows aging-related apoptosis, heart hypertrophy, and fibrosis, and it delays cardiac aging [23]. Autophagy removes aggregated proteins and damaged organelles, reduces reactive oxygen species (ROS), and alleviates oxidative stress. However, when the level of oxidative stress exceeds the limit of the body's protective mechanisms, the large amounts of ROS cause excessive self-digestion of the cellular components. The autophagic machinery is exhausted, resulting in the inhibition of autophagy and leading to cell death and aging [24].

In this study, we established an oxidative stress-induced aging model using D-galactose. D-galactose is converted into galactitol, which accumulates in the cell and induces the production of excessive ROS [25]. Following the treatment of primary cardiomyocytes with D-galactose for 48 h, the levels of intracellular ROS increased, accompanied by decreased autophagy. Oxidative stress is the main contributor to the cardiac aging processes. Autophagy is reduced in senescent cardiomyocytes, which could be attributed to the exhaustion caused by excessive oxidative stress. This finding is in line with that of a previous study on cardiac aging.

Autophagy is regulated by various signaling pathways during cardiac aging. Inducing autophagy is considered a potential therapeutic strategy for treating cardiac aging.

There are two protein complex forms of the mammalian target of rapamycin (mTOR): mTORC1 and mTORC2. In the mouse heart, mTORC1 activity increases with age. mTORC1 regulates cell growth, proliferation, survival, protein translation, ribosome genesis, autophagy, and other processes [26]. During cardiac aging, the key upstream regulatory pathway of mTORC1 is the AMPK/mTOR pathway.

An increase in the ratio of AMP to ATP activates AMP-activated protein kinase (AMPK), which negatively regulates MTORC1. AMPK activates and phosphorylates tuberous sclerosis 1/2 (TSC1/2), a downstream mTOR inhibitor, and Raptor, an mTORC1 inhibitor. AMPK directly phosphorylates ULK1 and Beclin1 to activate them [15]. In aging hearts, AMPK phosphorylation levels continuously decrease [27]. Chen et al. used exogenous hydrogen sulfide to stimulate senescence in H9C2 cells *in vitro* and aging mice *in vivo*. The expression of autophagy-related proteins, Beclin-1, LC3II, and ATG5 increased significantly. In addition, the levels of phosphorylated AMPK and P62 increased, while the level of phosphorylated mTOR decreased. Exogenous hydrogen sulfide induced autophagy by upregulating the AMPK/mTOR pathway in aging mice and senescent cardiomyocytes [28].

Sirtuins (SIRT) are a class of histone deacetylases with seven isoforms that influence cellular stress, apoptosis, and senescence. SIRT1 is the most studied protein in the sirtuin family. SIRT1 is crucial for autophagy and longevity [29]. Baicalein induces mitochondrial autophagy by modulating the SIRT1/AMPK/mTOR pathway. It delays Parkinson's disease, a major neurodegenerative disease. Therefore, we hypothesized that the SIRT1/AMPK/mTOR pathway regulates autophagy in aging hearts. In D-galactose-induced senescent cardiomyocytes, the levels of SIRT1 and phosphorylated AMPK decreased, however, phosphorylated mTOR expression increased. The SIRT1/AMPK/mTOR pathway is inhibited in cardiac aging, in line with depressed autophagy. SIRT1 gene knockdown using sirt1 siRNA, followed by D-galactosidase stimulation indicated that cardiomyocyte senescence and intracellular ROS levels were exacerbated in cardiomyocytes transfected with siSIRT1. Autophagy was further inhibited, phosphorylated AMPK levels decreased, and phosphorylated mTOR levels increased, suggesting that SIRT1/AMPK/mTOR can enhance autophagy to improve aging and attenuate oxidative stress in D-galactose-induced senescent cardiomyocytes. Our findings are consistent with those of Chen et al., suggesting that the SIRT1/AMPK/mTOR pathway can positively regulate autophagy to improve cardiac senescence and could be a target for developing therapeutics against cardiac senescence. We used primary rat cardiomyocytes, which are closer to the *in vivo* physiological conditions than cell lines. Therefore, the results were more reliable than those from the previous study.

The polyphenol compound, curcumin, extracted from turmeric, has various therapeutic uses in humans. It induces antioxidant, anti-inflammatory, anticancer, and antiaging effects [30]. Curcumin protects against cardiovascular diseases, such as cardiac hypertrophy, heart failure, and atherosclerosis. The role of curcumin in regulating apoptosis and autophagy is well-studied [31], including its role in reversing the aging process and reducing oxidative stress. Curcumin pretreatment for 24 h inhibits hydrogen peroxide-induced premature senescence in endothelial cells, decreased ROS production, and increased eNOS and NO production [32]. In diabetic cardiomyopathy, curcumin activates autophagy by enhancing the levels of AMPK and JNK1, subsequently alleviating apoptosis [33]. Isoproterenol-induced cardiac hypertrophy could be alleviated by curcumin by enhancing autophagy via AMPK/mTOR. Additionally, SIRT1 activation is linked to the protective effects [34].

Curcumin has been studied extensively. However, its effect on cardiac aging and the underlying mechanism of action remains unclear. Therefore, we aimed to explore the effect of curcumin on cardiac aging and its possible mechanism of action. Curcumin promoted autophagy and reduced intracellular ROS in a dose-dependent manner, thus improving cardiac aging. In addition, inhibiting SIRT1 gene expression indicated that curcumin promoted autophagy through the SIRT1/AMPK/mTOR pathway.

Curcumin ameliorates aging by promoting autophagy and reducing oxidative stress during oxidative stress-induced cardiac aging. These protective effects of curcumin in cardiac aging is consistent with the interaction between autophagy and oxidative stress. In addition, curcumin could be used as a potential pharmacological candidate for treating cardiac aging. Curcumin plays a cardioprotective role through the SIRT1/AMPK/mTOR pathway, suggesting that this pathway could be a potential target for developing future drugs.

However, this study has certain limitations. *In vivo* experiments should be conducted in the future.

## 5. Conclusions

In this paper, the experimental results confirmed that curcumin alleviated cardiac aging by promoting autophagy and reducing oxidative stress *in vivo*. The experimental results also revealed that curcumin acted as a cardioprotective agent via the SIRT1/AMPK/mTOR pathway.

## Figures and Tables

**Figure 1:** Curcumin inhibited D-galactose-induced senescence and decreased ROS in cardiomyocytes. (a) Primary neonatal rat cardiomyocytes were treated with D-gal (10 g/l). The suppression effect of curcumin on primary neonatal rat cardiomyocyte senescence shown by SA-*β*-galactosidase staining (*n* = 5). Scale bar: 100 *μ*m. (b) SA-*β*-galactosidase-positive cells. (c) Curcumin inhibited the expression of the senescence markers p53 and p16 in senescent cardiomyocytes, as observed using western blot (*n* = 5). (d) p53 expression. (e) p16 expression. (f) Curcumin reduces intracellular ROS levels in cardiomyocytes as observed using the DCFH-DA probe staining, *n* = 5, scale bar: 100 *μ*m. (g) Statistical results for ROS production.  ^*∗∗*^*P* < 0.01 vs. control.  ^#^*P* < 0.05,  ^#^ ^#^*P* < 0.01, vs. D-gal. The data are expressed as mean ± SEM.

**Figure 2:** Curcumin promoted autophagy in D-galactose-induced senescent cardiomyocytes. (a) Curcumin improved the ratio of LC3 II/I. Moreover, it attenuated P62 expression (*n* = 5). (b) Quantitation results of LC3 II/I. (c) Quantitation results of p62. (d) Representative images of mRFP -GFP-LC3 stain. Cardiomyocytes were transfected with the GFP-RFP-LC3 adenovirus for 24 h and exposed to D-gal (10 g/l) with different concentrations of curcumin for 48 h. The yellow dots represent autophagosomes, and the red dots indicate autolysosomes. We counted the GFP and mRFP dots. Three independent experiments were conducted. A total of 10 cells were scored in each experiment. Scale bars: 20 mm. (e) Quantification of relative LC3 dots was plotted.  ^*∗∗*^*P* < 0.01 vs. control.  ^#^*P* < 0.05,  ^#^ ^#^*P* < 0.01, vs. D-gal. The data are expressed as the mean ± SEM.

**Figure 3:** Curcumin enhanced the SIRT1-AMPK/mTOR signal pathway. (a) Representative western blot for SIRT1 p-AMPK and p-mTOR levels in cardiomyocyte lysates (*n* = 5). (b) Quantitation results of p-mTOR. (c) Quantitation results of SIRT1. (d). Quantitation results of p-AMPK.  ^*∗∗*^*P* < 0.01 vs. control.  ^#^*P* < 0.05,  ^#^ ^#^*P* < 0.01, vs. D-gal. The data are expressed as the mean ± SEM.

**Figure 4:** siSIRT1 blocked the antiaging and antioxidant effect of curcumin in D-galactose-induced senescent cardiomyocytes. (a) Representative SA-*β*-galactosidase staining images showing that SIRT1 knockdown inhibited the antiaging effects of curcumin in senescent cardiomyocytes, as observed through the increased number of SA-*β*-galactosidase positive cells (*n* = 5). Scale bar: 100 *μ*m. (b) Results of the statistics of SA-*β*-galactosidase staining. (c) Representative western blot of P53 and p16 (*n* = 5). (d) Quantitation results of p53. (e) Quantitation results of p16. (f) SIRT1 siRNA blocked the antioxidant effect of curcumin in D-galactose-induced senescent cardiomyocytes. Representative images of DCFH-DA staining indicated that ROS production in senescent cardiomyocytes is reduced because of the effect of curcumin (*n* = 5). Scale bar: 100 *μ*m. (g) Statistical results for ROS production.  ^#^*P* < 0.05,  ^#^ ^#^*P* < 0.01, vs. control siRNA. The data are expressed as the mean ± SEM.

**Figure 5:** siSIRT1 inhibited the promotion of autophagy by curcumin in D-galactose-induced senescent cardiomyocytes. (a) LC3 II/I and p62 levels indicated the suppression of the promoting autophagy effects of curcumin by sirt1 gene knockdown (*n* = 5). (b) The quantitation results of LC3 II/I. (c) The quantitation results of p62. (d) Representative images showed less autophagy because of the inhibition of siSIRT1-mediated knockdown, GFP-RFP-LC3 adenovirus transfected for 24 h: 50 *μ*m. (e) The quantification of relative LC3 points was plotted.  ^#^*P* < 0.05,  ^#^ ^#^*P* < 0.01, vs. control. The data are expressed as the mean ± SEM.

**Figure 6:** (a) Representative western blot of the levels of SIRT1 p-AMPK and p-mTOR. siSIRT1-mediated knockdown blocked the inducing effect of curcumin on the SIRT1/AMPK/mTOR pathway in cardiac aging (*n* = 5). (b) The quantitation results of SIRT1. (c) The quantitation results of p-AMPK. (d) The quantitation results of p-mTOR.  ^#^*P* < 0.05,  ^#^ ^#^*P* < 0.01, vs. control. The data are expressed as the mean ± SEM.

## Data Availability

The data used to support the findings of this study are included within the article.
